# Tumor glycolysis as a target for cancer therapy: progress and prospects

**DOI:** 10.1186/1476-4598-12-152

**Published:** 2013-12-03

**Authors:** Shanmugasundaram Ganapathy-Kanniappan, Jean-Francois H Geschwind

**Affiliations:** 1 Russell H Morgan Department of Radiology & Radiological Sciences, Division of Interventional Radiology, Johns Hopkins University School of Medicine, 600 N. Wolfe Street, Blalock Building 340, 21287 Baltimore, MD, USA; 2 Russell H. Morgan Department of Radiology and Radiological Sciences, Division of Vascular and Interventional Radiology, Sheikh Zayed Tower, Suite 7203, The Johns Hopkins Hospital, 1800 Orleans Street, 21287 Baltimore, MD, USA

**Keywords:** Glycolysis, Antiglycolytic agents, Cancer metabolism, Chemotherapy

## Abstract

Altered energy metabolism is a biochemical fingerprint of cancer cells that represents one of the “hallmarks of cancer”. This metabolic phenotype is characterized by preferential dependence on glycolysis (the process of conversion of glucose into pyruvate followed by lactate production) for energy production in an oxygen-independent manner. Although glycolysis is less efficient than oxidative phosphorylation in the net yield of adenosine triphosphate (ATP), cancer cells adapt to this mathematical disadvantage by increased glucose up-take, which in turn facilitates a higher rate of glycolysis. Apart from providing cellular energy, the metabolic intermediates of glycolysis also play a pivotal role in macromolecular biosynthesis, thus conferring selective advantage to cancer cells under diminished nutrient supply. Accumulating data also indicate that intracellular ATP is a critical determinant of chemoresistance. Under hypoxic conditions where glycolysis remains the predominant energy producing pathway sensitizing cancer cells would require intracellular depletion of ATP by inhibition of glycolysis. Together, the oncogenic regulation of glycolysis and multifaceted roles of glycolytic components underscore the biological significance of tumor glycolysis. Thus targeting glycolysis remains attractive for therapeutic intervention. Several preclinical investigations have indeed demonstrated the effectiveness of this therapeutic approach thereby supporting its scientific rationale. Recent reviews have provided a wealth of information on the biochemical targets of glycolysis and their inhibitors. The objective of this review is to present the most recent research on the cancer-specific role of glycolytic enzymes including their non-glycolytic functions in order to explore the potential for therapeutic opportunities. Further, we discuss the translational potential of emerging drug candidates in light of technical advances in treatment modalities such as image-guided targeted delivery of cancer therapeutics.

## Introduction

Glucose metabolism in cancer cells is primarily characterized by two major biochemical events: (i) increased glucose uptake and (ii) aerobic glycolysis, the process of conversion of glucose into pyruvate eventually resulting in the production of lactate (fermentation). The former has already been exploited clinically to diagnose cancer and assess tumor response through the utilization of radiolabeled glucose analog, ^18^Fluoro-deoxyglucose (FDG) in positron emission tomography (PET). PET imaging, combined with computed tomography (CT), plays an indispensable role in modern diagnostic oncology [1]. But it is the notion that tumor glycolysis could be used as a potential target for therapy that remain the most intriguing. The existence of a link between aerobic glycolysis (i.e. glycolysis in the presence of oxygen) and tumorigenesis has been known for several decades ever since the German scientist Otto Warburg proposed the “Warburg hypothesis” known as the “Warburg effect” [2,3]. Yet, the underlying mechanistic details pertinent to the causes and consequences of such metabolic phenotype remained unclear. Conceptual advances in the past decades have improved our understanding on the biological significance of tumor metabolism [4]. As a result, deregulated or altered energy metabolism has been recognized as one of the “hallmarks of cancer” [5].

It is increasingly evident that oncogenes and tumor suppressors regulate altered energy metabolism. Oncogenic mutations culminate in the up-regulation of glucose transporters (e.g. GLUT 1, GLUT 3) [6,7] thus facilitating increased glucose consumption by cancer cells, which in turn increases the rate of glucose metabolism. Conversely, the glycolytic/metabolic phenotype confers selective advantage to cancer cells by supporting uninterrupted growth. For example, a higher glycolytic rate in tumor cells has been shown to promote resistance to chemotherapeutics. In the cervical cancer cell line, HeLa for example, the enzyme pyruvate dehydrogenase kinase (PDK) isoforms PDK1 and PDK3 have been demonstrated to provide resistance to chemotherapeutics [8]. Similarly, in the colon carcinoma cell line, LoVo it has been demonstrated that increased aerobic lactate production (glycolysis) correlated with drug resistance [9]. Thus, interrupting or possibly disrupting tumor glycolysis will impact tumor growth by energy depletion as well as sensitization to therapeutics especially, in light of the recent reports that have elucidated cancer-specific advantages of aerobic glycolysis [10-13]. Several authors have delineated a wealth of information on the biochemical targets of glycolysis and their potent antagonists or inhibitors with promising anticancer effects (refer reviews [14-18]). Our goal in this review is to discuss the cancer-specific intricacies and advantages of glycolysis in the light of recent research underscoring the clinical relevance of targeting it for cancer therapy.

### Glycolysis in cancer

The fact that cancer cells express the glycolytic phenotype has long been known (refer review, [19]). However, until recently, the dependence on such a phenotype remained unclear. In an elegant report, Bonnet et al. [20] demonstrated that reversing the glycolytic phenotype to oxidative phosphorylation (OXPHOS) in cancer cells resulted in the induction of cell death. Further, when the mitochon-drial-K^+^ channel axis of cancer cells is suppressed, a mere restoration of mitochondrial-K^+^ channel function is sufficient to promote apoptosis. This report supports two major hypotheses, (i) reversal of the glycolytic phenotype to oxidative phosphorylation can promote cancer cell death and (ii) glycolysis can facilitate tumor growth despite a suppressed mitochondria-K^+^ channel axis.

Understandably, the metabolic switch from mitochondrial respiration to glycolysis during hypoxia (where oxidative phosphorylation will be inactive) as well as mitochondrial dysfunction [21,22] are critical for cancer cell growth. Yet, the presence of aerobic glycolysis under normoxic conditions in the context of functionally efficient mitochondria is also very intriguing. Mitochondrial impairment or defective oxidative phosphorylation is frequently found in cancer. It is known that mutations in mitochondrial DNA (mtDNA) affect the enzymes involved in OXPHOS, at least three enzymes from the TCA cycle, succinate dehydrogenase (SDH), fumarate dehydrogenase (FDH) and isocitrate dehydrogenase (IDH) (reviewed by Wallace [23]) whereas mitochondrial gene mutations in the nuclear DNA (nDNA) primarily affect the bioenergetics status of cancer cells (reviewed by Wallace [23]). These enzymatic mutations have been linked to several intrinsic pathways that together or independently can reprogram the metabolic circuitry of cancer cells. For example, SDH mutation results in the accumulation of succinate which in turn inhibits prolyl hydroxylase dehydroganse (PHD) eventually contributing for the stabilization of HIF-1α. This mechanism is sufficient to recognize the importance of HIF-1α’s role as an activator of aerobic glycolysis and lactate production. Thus it is clear that mitochondrial defect in cancer cells can cause a shift in energy metabolism.

On the other hand, cancer cells subjected to mtDNA gene mutations or deletions show reduced colony formation, growth rate and diminished tumorigenicity [24]. Based on this and similar reports, if impaired mitochondria were truly a “common cause of cancer growth” as proposed by Warburg, then it is difficult to explain the rapid proliferation, formation of metastases and chemoresistance typical of cancer cells. It could then be that such cancer cells harbor the functionally normal mitochondria from surrounding normal cells [25]. If this were the case, it could not support the theory that a mitochondrial defect is at the origin of “aerobic glycolysis or lactate production” as normal mitochondria (located in adjacent normal healthy cells) could compensate for the OXPHOS function. Nevertheless, a wealth of data indicate that a link between mitochondrial function and cancer progression exists, especially with the energy metabolism of cancer cells, although a distinctive step-wise mechanistic principle underlying the origin of cancer remains extremely controversial.

Recent investigations have shed light on the understanding of the benefits and selective advantages of aerobic glycolysis. Although glycolysis yields a lower amount of ATP compared to mitochondrial OXPHOS, several key benefits inherent in aerobic glycolysis drive cancer cells to favor glycolysis over mitochondrial oxidation [26]. First, the rate of glycolysis and turnover of glucose into lactic acid is accelerated thereby resulting in faster and greater ATP production. Pfeiffer et al. [27] have postulated that the high-rate but low yield ATP producing pathway (glycolysis) confer selective advantage under competition for shared energy sources, adding an evolutionary significance to glycolysis [28]. The rate of ATP production may be 100 times faster with glycolysis than with OXPHOS [29]. The low yield of ATP with glycolysis is however sufficient to meet intracellular demand. Rapidly dividing cells such as microorganisms (with a doubling time ranging from a few minutes to several hours) require ATP for proliferation whereas cancer cells with a comparatively longer doubling time (days rather than minutes) may require ATP primarily only for cell maintenance (rather than for proliferation). For all these reasons, the ATP formed through glycolysis is sufficient for cancer growth. It is therefore likely that the increased rate of ATP production resulting from glycolysis confers a selective growth advantage to cancer cells [30,31]. Second, in addition to ATP, cancer cells require further metabolic intermediates and precursors that are critical for the biosynthesis of macromolecules, the ultimate building blocks indispensable to increase the tumor mass during growth and proliferation [32]. The accumulation of glycolytic intermediates is known to promote the pentose phosphate pathway PPP resulting in the generation of NADPH and ribose-5-phosphate. Both, NADPH and ribose-5-phosphate are essential for the biosynthesis of lipids and nucleic acids. Lastly, the production of NADPH enables the cancer cells to maintain adequate levels of reduced forms of glutathione (GSH), a key non-enzymatic antioxidant. GSH plays a pivotal role in protecting cancer cells against antineoplastic agents by maintaining the redox status as well as by counteracting some of the effects from chemotherapeutic agents (reviewed [33,34]). In this context, under experimental conditions, Zhou et al. [28], have demonstrated that chemoresistant cell lines have elevated aerobic glycolysis indicating a biochemical link between resistance and glycolysis. Apart from the resistance to chemotherapeutics, aerobic glycolysis has also been implicated in resistance to radiotherapy. Indeed, Pitroda et al. [35] have demonstrated that regulation of glycolytic or energy metabolic pathway affects the sensitivity of tumor cells.

The PPP plays a pivotal role in macromolecular biosynthesis. Recent evidence indicates that it also contributes to therapeutic resistance as an antioxidant system to chemo- and radiation therapies [36]. Among several enzymes involved in the PPP, the transketolase (TKTL1) has gained increased attention owing to its involvement in cell survival under stress or starvation [37-39]. Other data also indicate that TKTL1 affects the chemosensitivity of cancer cells to drugs such as imatinib [40], cetuximab [41]. Thus it is evident that aerobic glycolysis in conjunction with the pentose shunt pathway provide multiple benefits to cancer cells such as promoting tumor progression and providing resistance to therapy. Hence, this key signature of cancer cells, tumor metabolism, particularly the tumor glycolysis, provides an ideal target for therapeutic intervention.

### Non-glycolytic functions of glycolytic enzymes and the metabolic intermediates

Many enzymes of the glycolytic pathway also play significant roles in several non-glycolytic processes that enable the cancer cells to meet other cellular demands. As shown in Figure 1, enzymes such as hexokinase II (HKII), glyceraldehyde-3-phosphate dehydrogenase (GAPDH), pyruvate kinase (PK)-M2 isoform and lactate dehydrogenase (LDH) are known to be involved in a number of subcellular functions including transcriptional regulation and phosphorylation of histones [42].

**Figure 1:** **Non-glycolytic functions of glycolytic enzymes and metabolic intermediates.** In the innermost circle, thick arrows represent enzymes and thin arrows indicate intermediate metabolites. The short arrows pointing towards the outer circle represent the non-glycolytic functions of corresponding enzymes/metabolites.

For example, the mitochondrial membrane-bound HKII antagonizes the proapoptotic machinery there by provides survival advantage to cancer cells [43,44]. In addition, HKII is also involved in transcriptional regulation, a functional property characteristic of nuclear proteins [42]. Similarly, GAPDH plays a crucial role in the maintenance of cellular redox balance as it catalyses the first step to produce NADH (extensively reviewed by Seidler [45]). It is also known that GAPDH plays a pivotal role in protecting the cells from free radical or ROS-mediated injury. As for the nuclear functions of GAPDH available reports indicate that GAPDH might be involved in both pro-apoptotic and oncogenic processes (Seidler, [46]). Its oncogenic role involves the indirect participation in nucleic acid binding properties of hepatitis viruses – a function that correlates with liver carcinogenesis [47]. What remains to be elucidated is the identification of the intracellular mechanism that directs the proapoptotic or oncogenic role of GAPDH. Next, PK-M2 is involved in the regulation of macromolecular biosynthesis (e.g. nucleic acid) [48] and multiple reports have established its role in tumor progression [49-51]. In addition to its involvement in biosynthesis, nuclear translocation of its phosphorylated form has been shown to promote the Warburg effect [52]. Several reports have indicated that PK-M2 strongly participates in diverse non-glycolytic functions [53]. PK-M2 acts as a kinase and phosphorylates histone H3 to favor tumorigenesis [54], as a nuclear protein it transactivates β-catenin [55], and as a phosphotyrosine binding protein it interacts with other proteins as well [56]. Evidence from gene silencing experiments demonstrate that the enzyme, LDH cooperates with Oct-4, a transcriptional factor, during gastric tumorigenesis. Silencing LDH abrogated tumorigenicity by Oct-4 down regulation (19). Thus many glycolytic enzymes participate or influence several non-metabolic functions.

As with glycolytic enzymes, some of the metabolic intermediates of glycolysis have also been associated with non-glycolytic pathways. For example, Fructose-1, 6 bisphosphate plays an anti-apoptotic role in cancer cells by maintaining the cytochrome C in a reduced, non-active state [57]. Similarly, pyruvate contributes to chemoresistance by over-expressing the p-glycoprotein [58]. The export and import of lactate (the product of pyruvate oxidation) is achieved through the transporters known as monocarboxylate transporters (MCTs). The non-glycolytic role of MCTs include the regulation of the CD147, a matrix metalloproteinase inducer, which increases the invasion and metastatic potential of cancer cells [59,60]. Collectively, these findings strongly suggest that many of the enzymes and metabolic intermediates of tumor glycolysis also play a key role beyond glycolysis, thereby facilitating the growth and survival of cancer cells.

Increasing evidences demonstrate that glycolytic enzymes translocate to different subcellular compartments where they can interact with subcellular structures to an appreciable degree resulting in significant differences in their primary and secondary functions (Figure 2). The enzyme HKII which catalyses the first rate-limiting step of glucose metabolism is located proximally to the mitochondria in order to facilitate the immediate utilization of ATP. Similarly, other glycolytic enzymes such as GAPDH and aldolase are anchored by actin filament-like structures located in close proximity to the segments of glycolysis taking place in the cytoplasm [61].

**Figure 2:** **Schematic showing the distribution of glycolytic enzymes in various subcellular compartments.** HKII is a cytoplasmic enzyme however its localization to mitochondrial membrane has been established. As for binding with tubulin or actin filaments existing data are strong enough to include only GAPDH and for other glycolytic enzymes it remains to be known. The nuclear translocation has been well documented for the enzymes GAPDH, LDH, PFKFB3 and PK-M2.

Whereas the necessity and significance of the association between glycolytic enzymes and cytoskeletal structures remains obscure, the nuclear functions of glycolytic enzymes are sufficiently documented. Indeed, one of the isoforms of phosphofructo kinase (PFK), the PFKFB3 impacts cancer cell proliferation by its nuclear translocation [62]. Similarly, the direct binding of GAPDH to telomeric DNA protects telomeres against chemotherapy-induced rapid degradation [63]. GAPDH also enhances the transcriptional activity of androgen receptors in prostate cancer cells [64]. Finally, the nuclear translocation of LDH modulates the functions of DNA polymerases alpha, delta and epsilon [65]. It is convincingly evident that glycolytic enzymes participate in several non-glycolytic processes at various subcellular locations including the mitochondrial-membrane, as well as nuclear and cytoplasmic compartments.

### Relevance for targeting glycolysis

A higher lactate level significantly correlates with tumor recurrence and the metastatic potential of tumors resulting in poor patient outcomes [66]. As lactate level indicates the prevalence of glycolytic phenotype targeting such tumors through antiglycolytic agents likely to be very effective. Lactate was originally thought to be an acidic molecule that must be exported from cancer cells to prevent deleterious intracellular acidification. Recently, different roles of lactate export/import have been implicated with some directly contributing to cancer survival and growth and others to the metabolism of normoxic cancer cells that do not produce or excrete lactic acid. In this way, a sort of “metabolic symbiosis” exists within the tumor [67]; the lactate produced and extruded by hyperglycolytic or hypoxic cancer cells is able to re-enter normoxic cancer cells and be utilized to generate energy through mitochondrial oxidation [68]. In the heterogeneous tumor microenvironment characteristic of many solid tumors where both normoxic and hypoxic conditions co-exist, (depending upon angiogenesis and their proximity to blood vessels), the described “give and take lactate” mechanism [69] would mutually benefit both the lactate-exporting cells and the surrounding lactate-importing cells. In addition, the presence of lactate within the tumor microenvironment, which causes extreme acidic conditions, enables the deactivation or even inactivation of several chemotherapeutic agents. This process of lactate export and import is achievable by the over-expression of MCTs (primarily the MCT1 and MCT4). Note that the MCTs are over expressed in most tumors [70]. The release of lactate occurs through MCT4, whereas its uptake occurs through MCT1 [71]. In mouse and human tumors, MCT1 was found to be the major transporter ensuring lactate uptake by oxidative tumor cells and MCT4 as a hypoxia-induced transporter involved in the removal of lactate from glycolytic cells. Interestingly, MCT1 was found in the tumor cells of vascularized area whereas MCT4 was consistently concentrated in hypoxic regions correlating well with their known respective functions.

Recently, using untransformed primary breast cells (HMEC) as controls, Hussien and Brooks [72] demonstrated that a significant correlation exists between the expression profile of MCT isoforms (MCT-1 and 4) and the abundance of LDH isoforms (LDH A and B) in breast cancer cell lines (MDA-MB231 and MCF-7). In the MCF-7 cell line MCT1 (export of lactate) is abundant and LDHA, which converts pyruvate to lactate, is upregulated. On the other hand in the MDA-MB-231 cells, MCT4 is over expressed (uptake of lactate to be converted back to pyruvate for utilization in TCA cycle), LDHB is abundant. Thus cancer cells organize their glycolytic phenotype in a programmed fashion in order to achieve maximum efficiency. Thus it is conceivable that inhibition of glycolysis could be effective in killing both glycolytic and “symbiotic” non-glycolytic tumor cells.

Multiple lines of evidences have established that a higher expression levels of GLUTs and of certain enzymes such as HKII, GAPDH, LDH and PFK-B is linked to malignant growth [73-75]. As discussed elsewhere, it is increasingly evident that the cancer specific up-regulation of glycolysis is regulated through oncogenes (e.g. c-myc, Akt). The oncogenic activation directly up-regulates glycolytic enzymes [76] and/or through the hypoxia induced HIF-1alpha activation, which is a characteristic of tumor microenvironment [77]. The later has been experimentally verified using 3D-*in vitro* models, where spheroid-formation resulted in the promotion of a central hypoxic area eventually leading to an increase in the glycolytic flux [78]. Akt, the serine/threonine kinase, is an oncogene that promotes cancer growth [79]. Akt activates aerobic glycolysis, importantly, renders cancer cells dependent on glycolysis for survival [80].

Coordinated networks involving signaling pathways enable cancer cells to detect and integrate the immediate environmental conditions to balance their anabolic and catabolic processes. The mammalian Target of Rapamycin (mTOR) represents such a pathway where the intracellular energy sensing molecule AMPK can impact the mTOR complex I (mTORC1) mechanism of activation to either delay or halt the energy consuming synthetic processes [81]. Such an adaptation involves mTORC1-mediated regulation of the expression of glycolytic enzymes through the activation of genes such as c-myc and HIF1-alpha [81-83]. In summary, as aerobic glycolysis plays a major role in molecular events associated with oncogenesis targeting it could be not only a relevant but also a viable anticancer strategy.

### Molecular targets and inhibitors of glycolysis

Figure 3 depicts major biochemical reactions of glycolysis along with the enzymes involved and the energy utilized or produced during the process with an emphasis on current molecular targets. The most important role of glycolysis is to consume glucose and convert it into energy in the form of ATP. The consumption of glucose is an active process, which relies on specific transporters known as GLUTs. These GLUTs are over-expressed in almost all cancer types and hence contribute to the increased glucose utilization that is characteristic of the glycolytic phenotype, a key signature of cancer. The entire process of glycolysis can be divided between a “preparatory phase” where energy is consumed and a “pay-off phase” where net energy is generated in the form of ATP and NADH.

**Figure 3:** **Diagram showing the two phases of glycolysis and the molecular targets currently exploited for potential therapeutic drug strategies.** Energy molecules such as ATP and NADH are highlighted in yellow, black arrows indicate consumption while red arrows indicate the energy release. The enzymes involved in respective reactions are abbreviated and encircled, where as the block symbol shows the targets exploited for drug development in preclinical investigations.

There are several approaches to disrupting glycolysis. Since cancer cells depend on increased utilization of glucose as compared to normal healthy cells, glucose deprivation could be an effective anticancer approach and possibly used as a cancer-preventive strategy. Indeed, carbohydrate-restricted diets to treat cancer patients have been reported to have therapeutic benefits [84].

An obvious direct approach would be to block the GLUTs, which would prevent glucose entry into the cancer cell and lead to total disruption of the glycolytic pathway. Several such compounds (e.g. Phloretin, WZB117, Fasentin) demonstrated anticancer effects in preclinical models [6,85]. However, selective blockade of GLUTs in tumor cells remains a critical challenge as GLUTs are ubiquitously expressed in all mammalian cells.

Another approach is to target the enzyme HKII that is responsible for the first step of glycolysis that converts glucose to glucose-6-phosphate. This enzyme plays a pivotal role in tumor glycolysis. First, it is a rate limiting step that provides direct feedback inhibition thereby preventing the consumption of cellular ATP in turn preserving precious energy within the cancer cell. Second, it has a low Km (high affinity) for glucose. This characteristic facilitates the initiation of glycolysis specifically in times of low serum glucose levels, and along with its subcellular localization, (bound to mitochondrial membrane) plays a pivotal role in the energy metabolism of cancer cells [86,87]. Lonidamine is an inhibitor of HKII and has completed phase III trial. However its clinical success has so far been impaired by significant pancreatic and hepatic toxicities [88]. Similarly, another glucose analog 2-deoxyglucose (2-DG) also showed promising anticancer effects in preclinical models [89]. However, later studies revealed that the principal mechanism underlying 2-DG’s anticancer effects vary [90,91]. Moreover, contrary to its widely believed anticancer effects, 2-DG was shown to activate pro-survival pathways in cancer cells [92]. In addition, hypoxic cells demonstrated chemoresistance against 2-DG [93]. Thus the success of 2-DG as a single agent for antiglycolytic therapy has been challenged. However, in combination treatments, 2-DG showed encouraging outcomes providing a new window of opportunity in combination therapy [94,95].

PFK catalyzes another rate-limiting step of glycolysis and is regulated by allosteric effectors and covalent modifications such as phosphorylation. It is activated by AMP and fructose 2,6-bisphosphate (F-2, 6-BP). An abundance of ATP inhibits the activity of PFK, presumably representing a regulatory mechanism. However, F-2, 6-BP has the capability to override the inhibitory effect of ATP, and to perpetuate uninterrupted glycolytic flux. Predictably, F-2, 6-BP is elevated in cancer cells [96]. It is regulated by the activity of a family of bi-functional enzymes including PFKFBs which is also up-regulated in cancer cells. As a result, specific inhibitors of PFKFB3 are being developed in several laboratories. Preliminary studies revealed promising anticancer effects [97] but further investigations are necessary to assess whether this approach could potentially be successful in the clinic.

An alternative promising therapeutic approach to date in terms of inhibiting tumor glycolysis has been targeting the enzyme GAPDH. In many ways the GAPDH reaction is unique because GAPDH catalyzes the very first step in which energy in the form of NADH is produced, the so-called “pay-off phase” (Figure 3). As such, GAPDH is truly the initiator of the “pay-off phase”. The first molecule produced during the “pay-off phase”, NADH, is critically involved in the regulation of intracellular ROS levels, and macromolecular biosynthetic processes. Thus, by producing NADH, GAPDH plays a pivotal role in the cellular redox balance. From a therapeutic point of view given the central role of GAPDH, it is conceivable that, apart from blocking glycolysis and ATP production, GAPDH inhibition would result in multipronged effects within the cancer cell. Inhibition of GAPDH triggers a cascade of events that eventually leads to cancer cell death. First, glucotrioses such as glyceraldehyde-3-phosphate and dihydroxy acetone phosphate accumulate within the cell since they cannot be metabolized. The partial degradation of these glucotrioses results in the formation of a cytotoxic metabolite, methylglyoxal. Normally, the methylglyoxal enters the glyoxalase system to be detoxified. However, in the presence of oxidative stress and GSH depletion secondary to the accumulation of ROS, the glyoxalase 1 (Glo1) activity diminishes leading to the accumulation of methylglyoxal which is directly cytotoxic. Under normal conditions, the methylglyoxal is detoxified by the Glo1 and Glo2 enzymes. But since the activity of both enzymes depends on the level of intracellular GSH, any oxidative stress and resulting increase in ROS level directly and swiftly affect the level of GSH, thus impacting the detoxification ability of methylglyoxal by Glo1 and Glo2 [98]. Inhibition of GAPDH therefore not only directly depletes ATP but also triggers a multipronged attack within the cell. Thus, inhibiting GAPDH not only affects tumor glycolysis (by blocking the most important energy producing step) but also provides an opportunity to exploit other cytotoxic mechanisms related to it.

Since GAPDH represents an attractive target for therapeutic intervention several inhibitors have already been tested for their efficacy in cell cultures as well as animal models [47]. One of the most promising of these inhibitors, the pyruvate analog 3-bromopyruvate (3-BrPA) has demonstrated profound potency in its ability to inhibit tumor glycolysis as well as cause massive depletion of intracellular ATP [99,100]. In addition, 3-BrPA shows utmost specificity and selectivity for GAPDH both *in vitro* in multiple cell lines and *in vivo* in numerous animal models of cancer [101,102]. By binding to GAPDH inside the cancer cells, 3-BrPA depletes ATP profoundly depriving the cancer cells of any energy [103,104]. As a result of its potent anticancer effects, 3-BrPA has recently entered the early phase of clinical trials (phase I).

PK catalyzes the conversion of phosphoenolpyruvate (PEP) to pyruvate, and generates ATP in the process. Among various isoforms, the M2 isoform has gained much attention due to its elevated expression in tumor cells. PK-M2 exists in either active or inactive forms. The activity of this isoform depends on its conformation (tetramer, dimer or monomeric form). PK-M2 is critical for aerobic glycolysis and tumor energy metabolism [49,105]. As with PFK, PK is also regulated by allosteric effectors and by phosphorylation, PK being specifically activated by fructose-1, 6-bisphosphate [106]. Several preclinical studies have shown that PK-M2 could represent a potential therapeutic target [107,108]. Consequently, strategies to develop small molecule inhibitors specific for PK-M2 are in progress. If proven successful in clinical trials, PK-M2 inhibitors could play a significant role in the treatment of cancer [109].

LDH catalyzes the final step in the glycolytic pathway that converts pyruvate into lactate. The intracellular accumulation of lactate is extremely detrimental as the abundance of lactate drastically lowers intracellular pH. The export of lactate into the extracellular space is therefore necessary. It takes place through an active process involving specific transporters known as MCTs. Among the described isoforms, MCT1 and MCT4 have been the subject of intense investigation due to their role in the import and export of lactate. FX11, an inhibitor of LDH depletes intracellular ATP levels, which in turn significantly increase oxidative stress resulting in tumor cell death [110]. Similarly, oxamate, another inhibitor of LDH sensitizes resistant cancer cells to chemotherapeutic agents [111]. Thus inhibition of LDH has demonstrated promising effects in preclinical investigations and its further progress depends on the outcome of clinical trials.

MCTs are the final port of entry for the lactate shuttle. Depending upon the isoform of MCT (1 or 4) the lactate could be either exported or imported [70]. A known MCT inhibitor, α-cyano-4-hydroxy-cinnamic acid, has been shown to affect tumor growth [112]. The principal mechanism underlying the MCT blockade-associated antitumorigenic effects involves intracellular trapping of lactate, which at a prolonged state will result in intracellular acidification causing cancer cell death. However, further studies are warranted to demonstrate the target specificity and therapeutic efficacy of such experimental agents in order to progress towards translation into the clinic.

## Conclusions and future directions

As discussed earlier, the reliance of cancer cells on the glycolytic pathway for their energy needs has been known for decades and has even been successfully exploited diagnostically (FDG-PET imaging) for many years. Yet, targeting this pathway for therapy has not been translated to the clinic. One of the major impediments is to overcome undesirable effects such as systemic toxicity. Plausibly, this is due to the ubiquitous nature of the enzymes of glucose metabolism including glycolysis. But in all fairness, systemic toxicity is a major impediment to clinical progress of any anticancer agent, not just those targeting tumor glycolysis. The emergence of the concept of selective targeting with targeted delivery has provided an additional option to circumvent the problem of systemic toxicity. In the last few years, there has been growing interest in revisiting this approach. This strategy employs the use of image-guidance to deliver the drug where it is required, i.e. in the vicinity of the tumor. Recent advances in imaging technology allow for such precise targeting of tumors, be it directly intra-tumorally or intraarterially where the blood supply to the tumor can be exploited [113]. Such therapeutic approaches provide a unique dual advantage in evading systemic toxicity while improving the potency of the drug [114-116]. However, these approaches are only effective in treating localized disease (to the liver for example) but not for widely metastatic cancers.

Certainly, the scientific rationale for targeting tumor glycolysis is clearly sound and logical. It is based on the fact that tumor glycolysis is a true signature of cancer cells. A number of drug candidates have been tested mostly pre-clinically with mixed success. But some have been extremely promising and are about to enter the clinical arena. One of the keys to clinical success will reside in our ability to develop glycolytic inhibitors with a very high specificity for the molecular target. Recently, Birsoy et al. [117] demonstrated that selective targeting of cancer cells could be achieved if anticancer agents or toxic molecules utilize a mechanism specific for cancer, (such as 3-BrPA that enters cells through MCTs which in turn are upregulated in cancer).

Antiglycolytic agents may provide an additional line of attack in combination therapy. Combining chemotherapeutic drugs and glycolytic inhibitors have already been demonstrated to be promising strategy to overcome drug resistance in cancer. Since tumor glycolysis also plays a significant role in chemoresistance of cancer cells glycolytic inhibitors therefore have the potential to sensitize tumor cells and to improve the outcome of conventional chemotherapy. Such combination therapies have yielded better results in preclinical models. For example, the use of chemotherapeutic agents (adriamycin or paclitaxel) or radiation therapy resulted in improved efficacy, when applied after sensitizing tumor cells with 2-DG, a HKII inhibitor [94,95]. Similarly, several combination studies with the glycolytic inhibitor, 3-BrPA (that primarily targets GAPDH) have demonstrated superior efficacy [118-120]. Thus the combinatorial therapeutic approach remains a viable alternative for treating even resistant phenotypes.

The inhibition of glycolysis can also transform tumor cells into forms that are susceptible or sensitive to immunotherapy, thus opening a new window of opportunity for immunotherapy [121]. In summary, targeting tumor glycolysis is scientifically sound opening the door for a few emerging therapeutic options. Some are about to be tested comprehensively in the clinic. Only then will we know whether the potential exists for the birth of a true viable new class of anti-cancer agents.

## Abbreviations

3-BrPA: 3-bromopyruvate; GLUT: Glucose transporters; HKII: Hexokinase II; GAPDH: Glycerladehyde-3-phosphate dehydrogenase; PFK: Phospho fructo kinase; PFKFB: 6-phosphofructo-2-kinase/fructose-2, 6-bisphosphatases; PK: Pyruvate kinase; LDH: Lactate dehydrogenase; PK-M2: Pyruvate kinase M2; MCT: Monocarboxylate transporters.

## Competing interest

Dr. Geschwind is the founder of Presciencelabs LLC, a biotech firm currently developing the pyruvate analog 3-bromopyruvate (3-BrPA) for clinical use in liver cancer.

## Authors’ contributions

Both authors wrote and approved the manuscript.

## References

[B1] BomanjiJBCostaDCEllPJClinical role of positron emission tomography in oncologyLancet Oncol20012315716410.1016/S1470-2045(00)00257-611902566

[B2] WarburgOOn the origin of cancer cellsScience195612331913093140036–8075 (Print)10.1126/science.123.3191.30913298683

[B3] WarburgOOn respiratory impairment in cancer cellsScience19561243215269270PMID- 13471593 OWN - NLM STAT- MEDLINE (0036–8075 (Print))13351639

[B4] GeschwindJFGeorgiadesCSKoYHPedersenPLRecently elucidated energy catabolism pathways provide opportunities for novel treatments in hepatocellular carcinomaExpert Rev Anticancer Ther20044344945710.1586/14737140.4.3.44915161443

[B5] HanahanDWeinbergRAHallmarks of cancer: the next generationCell2011144564667410.1016/j.cell.2011.02.01321376230

[B6] MachedaMLRogersSBestJDMolecular and cellular regulation of glucose transporter (GLUT) proteins in cancerJ Cell Physiol2005202365466210.1002/jcp.2016615389572

[B7] PelicanoHMartinDSXuRHHuangPGlycolysis inhibition for anticancer treatmentOncogene200625344633464610.1038/sj.onc.120959716892078

[B8] LuCWLinSCChenKFLaiYYTsaiSJInduction of pyruvate dehydrogenase kinase-3 by hypoxia-inducible factor-1 promotes metabolic switch and drug resistanceJ Biol Chem200828342281062811410.1074/jbc.M80350820018718909PMC2661383

[B9] FanciulliMBrunoTGiovannelliAGentileFPDi PadovaMRubiuOFloridiAEnergy metabolism of human LoVo colon carcinoma cells: correlation to drug resistance and influence of lonidamineClin Cancer Res2000641590159710778993

[B10] HsuPPSabatiniDMCancer cell metabolism: Warburg and beyondCell2008134570370710.1016/j.cell.2008.08.02118775299

[B11] DangCVHamakerMSunPLeAGaoPTherapeutic targeting of cancer cell metabolismJ Mol Med201189320521210.1007/s00109-011-0730-x21301795PMC3345191

[B12] BirsoyKSabatiniDMPossematoRUntuning the tumor metabolic machine: targeting cancer metabolism: a bedside lessonNat Med20121871022102310.1038/nm.287022772555

[B13] DangCVLinks between metabolism and cancerGenes Dev201226987789010.1101/gad.189365.11222549953PMC3347786

[B14] GranchiCMinutoloFAnticancer agents that counteract tumor glycolysisChem Med Chem2012781318135010.1002/cmdc.20120017622684868PMC3516916

[B15] WardPSThompsonCBMetabolic reprogramming: a cancer hallmark even warburg did not anticipateCancer Cell201221329730810.1016/j.ccr.2012.02.01422439925PMC3311998

[B16] Cuperlovic-CulfMCulfASTouaibiaMLefortNTargeting the latest hallmark of cancer: another attempt at ‘magic bullet’ drugs targeting cancers’ metabolic phenotypeFuture Oncol20128101315133010.2217/fon.12.12123130930

[B17] ZhaoYButlerEBTanMTargeting cellular metabolism to improve cancer therapeuticsCell Death Dis20134e53210.1038/cddis.2013.6023470539PMC3613838

[B18] JangMKimSSLeeJCancer cell metabolism: implications for therapeutic targetsExp Mol Med201345e4510.1038/emm.2013.8524091747PMC3809361

[B19] ZhangYYangJMAltered energy metabolism in cancer: a unique opportunity for therapeutic interventionCancer Biol Ther2013142818910.4161/cbt.2295823192270PMC3572003

[B20] BonnetSArcherSLAllalunis-TurnerJHaromyABeaulieuCThompsonRLeeCTLopaschukGDPuttaguntaLBonnetSHarryGHashimotoKPorterCJAndradeMAThebaudBMichelakisEDA mitochondria-K + channel axis is suppressed in cancer and its normalization promotes apoptosis and inhibits cancer growthCancer Cell2007111375110.1016/j.ccr.2006.10.02017222789

[B21] HuYLuWChenGWangPChenZZhouYOgasawaraMTrachoothamDFengLPelicanoHChiaoPJKeatingMJGarcia-ManeroGHuangPK-ras(G12V) transformation leads to mitochondrial dysfunction and a metabolic switch from oxidative phosphorylation to glycolysisCell Res201222239941210.1038/cr.2011.14521876558PMC3257361

[B22] LuWHuYChenGChenZZhangHWangFFengLPelicanoHWangHKeatingMJLiuJMcKeehanWWangHLuoYHuangPNovel role of NOX in supporting aerobic glycolysis in cancer cells with mitochondrial dysfunction and as a potential target for cancer therapyPLoS Biol2012105e100132610.1371/journal.pbio.100132622589701PMC3348157

[B23] WallaceDCMitochondria and cancerNat Rev Cancer2012121068569810.1038/nrc336523001348PMC4371788

[B24] CavalliLRVarella-GarciaMLiangBCDiminished tumorigenic phenotype after depletion of mitochondrial DNACell Growth Differ1997811118911989372242

[B25] KingMPAttardiGHuman cells lacking mtDNA: repopulation with exogenous mitochondria by complementationScience1989246492950050310.1126/science.28144772814477

[B26] de SouzaACJustoGZde AraujoDRCavagisADDefining the molecular basis of tumor metabolism: a continuing challenge since Warburg's discoveryCell Physiol Biochem201128577179210.1159/00033579222178931

[B27] PfeifferTSchusterSBonhoefferSCooperation and competition in the evolution of ATP-producing pathwaysScience2001292551650450710.1126/science.105807911283355

[B28] ZhouYTozziFChenJFanFXiaLWangJGaoGZhangAXiaXBrasherHWidgerWEllisLMWeihuaZIntracellular ATP levels are a pivotal determinant of chemoresistance in colon cancer cellsCancer Res201272130431410.1158/0008-5472.CAN-11-167422084398PMC3601736

[B29] LocasaleJWCantleyLCAltered metabolism in cancerBMC Biol201088810.1186/1741-7007-8-8820598111PMC2892450

[B30] GatenbyRAGilliesRJWhy do cancers have high aerobic glycolysis?Nat Rev Cancer200441189189910.1038/nrc147815516961

[B31] LuntSYVander HeidenMGAerobic glycolysis: meeting the metabolic requirements of cell proliferationAnnu Rev Cell Dev Biol20112744146410.1146/annurev-cellbio-092910-15423721985671

[B32] DeberardinisRJSayedNDitsworthDThompsonCBBrick by brick: metabolism and tumor cell growthCurr Opin Genet Dev2008181546110.1016/j.gde.2008.02.00318387799PMC2476215

[B33] BackosDSFranklinCCReiganPThe role of glutathione in brain tumor drug resistanceBiochem Pharmacol20128381005101210.1016/j.bcp.2011.11.01622138445

[B34] TraversoNRicciarelliRNittiMMarengoBFurfaroALPronzatoMAMarinariUMDomenicottiCRole of glutathione in cancer progression and chemoresistanceOxid Med Cell Longev201320139729132376686510.1155/2013/972913PMC3673338

[B35] PitrodaSPWakimBTSoodRFBeveridgeMGBeckettMAMacDermedDMWeichselbaumRRKhodarevNNSTAT1-dependent expression of energy metabolic pathways links tumour growth and radioresistance to the Warburg effectBMC Med200976810.1186/1741-7015-7-6819891767PMC2780454

[B36] RigantiCGazzanoEPolimeniMAldieriEGhigoDThe pentose phosphate pathway: an antioxidant defense and a crossroad in tumor cell fateFree Radic Biol Med201253342143610.1016/j.freeradbiomed.2012.05.00622580150

[B37] XuXZur HausenACoyJFLocheltMTransketolase-like protein 1 (TKTL1) is required for rapid cell growth and full viability of human tumor cellsInt J Cancer200912461330133710.1002/ijc.2407819065656

[B38] SunWLiuYGlazerCAShaoCBhanSDemokanSZhaoMRudekMAHaPKCalifanoJATKTL1 is activated by promoter hypomethylation and contributes to head and neck squamous cell carcinoma carcinogenesis through increased aerobic glycolysis and HIF1alpha stabilizationClin Cancer Res201016385786610.1158/1078-0432.CCR-09-260420103683PMC2824550

[B39] WankaCSteinbachJPRiegerJTp53-induced glycolysis and apoptosis regulator (TIGAR) protects glioma cells from starvation-induced cell death by up-regulating respiration and improving cellular redox homeostasisJ Biol Chem201228740334363344610.1074/jbc.M112.38457822887998PMC3460445

[B40] ZhaoFMancusoABuiTVTongXGruberJJSwiderCRSanchezPVLumJJSayedNMeloJVPerlAECarrollMTuttleSWThompsonCBImatinib resistance associated with BCR-ABL upregulation is dependent on HIF-1alpha-induced metabolic reprogramingOncogene201029202962297210.1038/onc.2010.6720228846PMC2874611

[B41] MonteleoneFRosaRVitaleMD'AmbrosioCSuccoioMFormisanoLNappiLRomanoMFScaloniATortoraGBiancoRZambranoNIncreased anaerobic metabolism is a distinctive signature in a colorectal cancer cellular model of resistance to antiepidermal growth factor receptor antibodyProteomics201313586687710.1002/pmic.20120030323281225

[B42] KimJWDangCVMultifaceted roles of glycolytic enzymesTrends Biochem Sci200530314215010.1016/j.tibs.2005.01.00515752986

[B43] PastorinoJGShulgaNHoekJBMitochondrial binding of hexokinase II inhibits Bax-induced cytochrome c release and apoptosisJ Biol Chem200227797610761810.1074/jbc.M10995020011751859

[B44] MajewskiNNogueiraVBhaskarPCoyPESkeenJEGottlobKChandelNSThompsonCBRobeyRBHayNHexokinase-mitochondria interaction mediated by Akt is required to inhibit apoptosis in the presence or absence of Bax and BakMol Cell200416581983010.1016/j.molcel.2004.11.01415574336

[B45] SeidlerNWGAPDH and intermediary metabolismAdv Exp Med Biol2013985375910.1007/978-94-007-4716-6_222851446

[B46] SeidlerNWBasic biology of GAPDHAdv Exp Med Biol201398513610.1007/978-94-007-4716-6_122851445

[B47] Ganapathy-KanniappanSKunjithapathamRGeschwindJFGlyceraldehyde-3-phosphate dehydrogenase: a promising target for molecular therapy in hepatocellular carcinomaOncotarget2012399409532296448810.18632/oncotarget.623PMC3660062

[B48] WuSLeHDual roles of PKM2 in cancer metabolismActa Biochim Biophys Sin (Shanghai)2013451273510.1093/abbs/gms10623212076

[B49] ChristofkHRVander HeidenMGHarrisMHRamanathanAGersztenREWeiRFlemingMDSchreiberSLCantleyLCThe M2 splice isoform of pyruvate kinase is important for cancer metabolism and tumour growthNature2008452718423023310.1038/nature0673418337823

[B50] LuoWSemenzaGLEmerging roles of PKM2 in cell metabolism and cancer progressionTrends Endocrinol Metab2012231156056610.1016/j.tem.2012.06.01022824010PMC3466350

[B51] LuoWSemenzaGLPyruvate kinase M2 regulates glucose metabolism by functioning as a coactivator for hypoxia-inducible factor 1 in cancer cellsOncotarget2011275515562170931510.18632/oncotarget.299PMC3248177

[B52] YangWZhengYXiaYJiHChenXGuoFLyssiotisCAAldapeKCantleyLCLuZERK1/2-dependent phosphorylation and nuclear translocation of PKM2 promotes the Warburg effectNat Cell Biol201214121295130410.1038/ncb262923178880PMC3511602

[B53] FilippFVCancer metabolism meets systems biology: Pyruvate kinase isoform PKM2 is a metabolic master regulatorJ Carcinog2013121410.4103/1477-3163.11542323961261PMC3746496

[B54] YangWXiaYHawkeDLiXLiangJXingDAldapeKHunterTAlfred YungWKLuZPKM2 phosphorylates histone H3 and promotes gene transcription and tumorigenesisCell2012150468569610.1016/j.cell.2012.07.01822901803PMC3431020

[B55] YangWXiaYJiHZhengYLiangJHuangWGaoXAldapeKLuZNuclear PKM2 regulates beta-catenin transactivation upon EGFR activationNature201148073751181222205698810.1038/nature10598PMC3235705

[B56] ChristofkHRVander HeidenMGWuNAsaraJMCantleyLCPyruvate kinase M2 is a phosphotyrosine-binding proteinNature2008452718418118610.1038/nature0666718337815

[B57] Diaz-RuizRAveretNAraizaDPinsonBUribe-CarvajalSDevinARigouletMMitochondrial oxidative phosphorylation is regulated by fructose 1,6-bisphosphate. A possible role in Crabtree effect induction?J Biol Chem200828340269482695510.1074/jbc.M80040820018682403

[B58] WartenbergMRichterMDatchevAGuntherSMilosevicNBekhiteMMFigullaHRAranJMPetrizJSauerHGlycolytic pyruvate regulates P-Glycoprotein expression in multicellular tumor spheroids via modulation of the intracellular redox stateJ Cell Biochem201010924344461995019910.1002/jcb.22422

[B59] Pertega-GomesNVizcainoJRMiranda-GoncalvesVPinheiroCSilvaJPereiraHMonteiroPHenriqueRMReisRMLopesCBaltazarFMonocarboxylate transporter 4 (MCT4) and CD147 overexpression is associated with poor prognosis in prostate cancerBMC Cancer20111131210.1186/1471-2407-11-31221787388PMC3157459

[B60] IzumiHTakahashiMUramotoHNakayamaYOyamaTWangKYSasaguriYNishizawaSKohnoKMonocarboxylate transporters 1 and 4 are involved in the invasion activity of human lung cancer cellsCancer Sci201110251007101310.1111/j.1349-7006.2011.01908.x21306479

[B61] MastersCCellular differentiation and the microcompartmentation of glycolysisMech Ageing Dev1991611112210.1016/0047-6374(91)90003-I1779698

[B62] YalcinAClemBFSimmonsALaneANelsonKClemALBrockESiowDWattenbergBTelangSChesneyJNuclear targeting of 6-phosphofructo-2-kinase (PFKFB3) increases proliferation via cyclin-dependent kinasesJ Biol Chem200928436242232423210.1074/jbc.M109.01681619473963PMC2782016

[B63] DemarseNAPonnusamySSpicerEKApohanEBaatzJEOgretmenBDaviesCDirect binding of glyceraldehyde 3-phosphate dehydrogenase to telomeric DNA protects telomeres against chemotherapy-induced rapid degradationJ Mol Biol2009394478980310.1016/j.jmb.2009.09.06219800890PMC2789664

[B64] HaradaNYasunagaRHigashimuraYYamajiRFujimotoKMossJInuiHNakanoYGlyceraldehyde-3-phosphate dehydrogenase enhances transcriptional activity of androgen receptor in prostate cancer cellsJ Biol Chem200728231226512266110.1074/jbc.M61072420017553795

[B65] PopandaOFoxGThielmannHWModulation of DNA polymerases alpha, delta and epsilon by lactate dehydrogenase and 3-phosphoglycerate kinaseBiochim Biophys Acta19981397110211710.1016/S0167-4781(97)00229-79545551

[B66] WalentaSWetterlingMLehrkeMSchwickertGSundforKRofstadEKMueller-KlieserWHigh lactate levels predict likelihood of metastases, tumor recurrence, and restricted patient survival in human cervical cancersCancer Res200060491692110706105

[B67] SonveauxPVegranFSchroederTWerginMCVerraxJRabbaniZNDe SaedeleerCJKennedyKMDiepartCJordanBFKelleyMJGallezBWahlMLFeronODewhirstMWTargeting lactate-fueled respiration selectively kills hypoxic tumor cells in miceJ Clin Invest200811812393039421903366310.1172/JCI36843PMC2582933

[B68] DraouiNFeronOLactate shuttles at a glance: from physiological paradigms to anti-cancer treatmentsDis Model Mech20114672773210.1242/dmm.00772422065843PMC3209642

[B69] SemenzaGLTumor metabolism: cancer cells give and take lactateJ Clin Invest200811812383538371903365210.1172/JCI37373PMC2582934

[B70] PinheiroCLongatto-FilhoAAzevedo-SilvaJCasalMSchmittFCBaltazarFRole of monocarboxylate transporters in human cancers: state of the artJ Bioenerg Biomembr201244112713910.1007/s10863-012-9428-122407107

[B71] FeronOPyruvate into lactate and back: from the Warburg effect to symbiotic energy fuel exchange in cancer cellsRadiother Oncol200992332933310.1016/j.radonc.2009.06.02519604589

[B72] HussienRBrooksGAMitochondrial and plasma membrane lactate transporter and lactate dehydrogenase isoform expression in breast cancer cell linesPhysiol Genomics201143525526410.1152/physiolgenomics.00177.201021177384PMC3068517

[B73] Hugo-WissemannDAnundiILauchartWViebahnRde GrootHDifferences in glycolytic capacity and hypoxia tolerance between hepatoma cells and hepatocytesHepatology199113229730310.1002/hep.18401302151847350

[B74] MikuriyaKKuramitsuYRyozawaSFujimotoMMoriSOkaMHamanoKOkitaKSakaidaINakamuraKExpression of glycolytic enzymes is increased in pancreatic cancerous tissues as evidenced by proteomic profiling by two-dimensional electrophoresis and liquid chromatography-mass spectrometry/mass spectrometryInt J Oncol200730484985517332923

[B75] YehCSWangJYChungFYLeeSCHuangMYKuoCWYangMJLinSRSignificance of the glycolytic pathway and glycolysis related-genes in tumorigenesis of human colorectal cancersOncol Rep2008191819118097579

[B76] RimpiSNilssonJAMetabolic enzymes regulated by the Myc oncogene are possible targets for chemotherapy or chemopreventionBiochem Soc Trans200735Pt 23053101737126610.1042/BST0350305

[B77] RobeyIFLienADWelshSJBaggettBKGilliesRJHypoxia-inducible factor-1alpha and the glycolytic phenotype in tumorsNeoplasia20057432433010.1593/neo.0443015967109PMC1501147

[B78] Rodriguez-EnriquezSGallardo-PerezJCAviles-SalasAMarin-HernandezACarreno-FuentesLMaldonado-LagunasVMoreno-SanchezREnergy metabolism transition in multi-cellular human tumor spheroidsJ Cell Physiol2008216118919710.1002/jcp.2139218264981

[B79] VivancoISawyersCLThe phosphatidylinositol 3-Kinase AKT pathway in human cancerNat Rev Cancer20022748950110.1038/nrc83912094235

[B80] ElstromRLBauerDEBuzzaiMKarnauskasRHarrisMHPlasDRZhuangHCinalliRMAlaviARudinCMThompsonCBAkt stimulates aerobic glycolysis in cancer cellsCancer Res200464113892389910.1158/0008-5472.CAN-03-290415172999

[B81] CsibiABlenisJAppetite for destruction: the inhibition of glycolysis as a therapy for tuberous sclerosis complex-related tumorsBMC Biol201196910.1186/1741-7007-9-6922018140PMC3198763

[B82] JiangXKenersonHAicherLMiyaokaREaryJBisslerJYeungRSThe tuberous sclerosis complex regulates trafficking of glucose transporters and glucose uptakeAm J Pathol200817261748175610.2353/ajpath.2008.07095818511518PMC2408433

[B83] DuvelKYeciesJLMenonSRamanPLipovskyAISouzaALTriantafellowEMaQGorskiRCleaverSVander HeidenMGMacKeiganJPFinanPMClishCBMurphyLOManningBDActivation of a metabolic gene regulatory network downstream of mTOR complex 1Mol Cell201039217118310.1016/j.molcel.2010.06.02220670887PMC2946786

[B84] KlementRJKammererUIs there a role for carbohydrate restriction in the treatment and prevention of cancer?Nutr Metab (Lond)201187510.1186/1743-7075-8-7522029671PMC3267662

[B85] LiuYCaoYZhangWBergmeierSQianYAkbarHColvinRDingJTongLWuSHinesJChenXA small-molecule inhibitor of glucose transporter 1 downregulates glycolysis, induces cell-cycle arrest, and inhibits cancer cell growth in vitro and in vivoMol Cancer Ther20121181672168210.1158/1535-7163.MCT-12-013122689530

[B86] MathupalaSPKoYHPedersenPLHexokinase II: cancer's double-edged sword acting as both facilitator and gatekeeper of malignancy when bound to mitochondriaOncogene200625344777478610.1038/sj.onc.120960316892090PMC3385868

[B87] MathupalaSPKoYHPedersenPLHexokinase-2 bound to mitochondria: cancer’s stygian link to the “Warburg Effect” and a pivotal target for effective therapySemin Cancer Biol2009191172410.1016/j.semcancer.2008.11.00619101634PMC2714668

[B88] PriceGSPageRLRiviereJEClineJMThrallDEPharmacokinetics and toxicity of oral and intravenous lonidamine in dogsCancer Chemother Pharmacol199638212913510.1007/s0028000504608616902

[B89] MaherJCKrishanALampidisTJGreater cell cycle inhibition and cytotoxicity induced by 2-deoxy-D-glucose in tumor cells treated under hypoxic vs aerobic conditionsCancer Chemother Pharmacol200453211612210.1007/s00280-003-0724-714605866

[B90] KurtogluMGaoNShangJMaherJCLehrmanMAWangpaichitrMSavarajNLaneANLampidisTJUnder normoxia, 2-deoxy-D-glucose elicits cell death in select tumor types not by inhibition of glycolysis but by interfering with N-linked glycosylationMol Cancer Ther20076113049305810.1158/1535-7163.MCT-07-031018025288

[B91] ZhongDLiuXSchafer-HalesKMarcusAIKhuriFRSunSYZhouW2-Deoxyglucose induces Akt phosphorylation via a mechanism independent of LKB1/AMP-activated protein kinase signaling activation or glycolysis inhibitionMol Cancer Ther20087480981710.1158/1535-7163.MCT-07-055918413794

[B92] ZhongDXiongLLiuTLiuXLiuXChenJSunSYKhuriFRZongYZhouQZhouWThe glycolytic inhibitor 2-deoxyglucose activates multiple prosurvival pathways through IGF1RJ Biol Chem200928435232252323310.1074/jbc.M109.00528019574224PMC2749096

[B93] MaherJCWangpaichitrMSavarajNKurtogluMLampidisTJHypoxia-inducible factor-1 confers resistance to the glycolytic inhibitor 2-deoxy-D-glucoseMol Cancer Ther20076273274110.1158/1535-7163.MCT-06-040717308069

[B94] MaschekGSavarajNPriebeWBraunschweigerPHamiltonKTidmarshGFDe YoungLRLampidisTJ2-deoxy-D-glucose increases the efficacy of adriamycin and paclitaxel in human osteosarcoma and non-small cell lung cancers in vivoCancer Res2004641313410.1158/0008-5472.CAN-03-329414729604

[B95] DwarakanathBJainVTargeting glucose metabolism with 2-deoxy-D-glucose for improving cancer therapyFuture Oncol20095558158510.2217/fon.09.4419519197

[B96] ChesneyJ6-Phosphofructo-2-Kinase/fructose-2,6-Bisphosphatase and Tumor Cell GlycolysisCurr Opin Clin Nutr Metab Care20069553553910.1097/01.mco.0000241661.15514.fb16912547

[B97] ClemBTelangSClemAYalcinAMeierJSimmonsARaskuMAArumugamSDeanWLEatonJLaneATrentJOChesneyJSmall-molecule inhibition of 6-phosphofructo-2-kinase activity suppresses glycolytic flux and tumor growthMol Cancer Ther20087111012010.1158/1535-7163.MCT-07-048218202014

[B98] ThornalleyPJRabbaniNGlyoxalase in tumourigenesis and multidrug resistanceSemin Cell Dev Biol201122331832510.1016/j.semcdb.2011.02.00621315826

[B99] KoYHSmithBLWangYPomperMGRiniDATorbensonMSHullihenJPedersenPLAdvanced cancers: eradication in all cases using 3-bromopyruvate therapy to deplete ATPBiochem Biophys Res Commun2004324126927510.1016/j.bbrc.2004.09.04715465013

[B100] PedersenPLThe cancer cell's “power plants” as promising therapeutic targets: an overviewJ Bioenerg Biomembr200739111210.1007/s10863-007-9070-517404823

[B101] Ganapathy-KanniappanSValiMKunjithapathamRBuijsMSyedLHRaoPPOtaSKwakBKLoffroyRGeschwindJF3-Bromopyruvate: a New Targeted Antiglycolytic Agent and a Promise for Cancer TherapyCurr Pharm Biotechnol201011551051710.2174/13892011079159142720420565

[B102] Ganapathy-KanniappanSKunjithapathamRGeschwindJFAnticancer efficacy of the metabolic blocker 3-bromopyruvate: specific molecular targetingAnticancer Res2013331132023267123

[B103] Ganapathy-KanniappanSGeschwindJFKunjithapathamRBuijsMVossenJATchernyshyovIColeRNSyedLHRaoPPOtaSValiMGlyceraldehyde-3-phosphate dehydrogenase (GAPDH) is pyruvylated during 3-bromopyruvate mediated cancer cell deathAnticancer Res200929124909491820044597PMC3743725

[B104] Pereira da SilvaAPEl-BachaTKyawNdos SantosRSda-SilvaWSAlmeidaFCDa PoianATGalinaAInhibition of energy-producing pathways of HepG2 cells by 3-bromopyruvateBiochem J2009417371772610.1042/BJ2008080518945211

[B105] SpodenGAMazurekSMorandellDBacherNAusserlechnerMJJansen-DurrPEigenbrodtEZwerschkeWIsotype-specific inhibitors of the glycolytic key regulator pyruvate kinase subtype M2 moderately decelerate tumor cell proliferationInt J Cancer2008123231232110.1002/ijc.2351218425820

[B106] DombrauckasJDSantarsieroBDMesecarADStructural basis for tumor pyruvate kinase M2 allosteric regulation and catalysisBiochemistry200544279417942910.1021/bi047492315996096

[B107] ChenJXieJJiangZWangBWangYHuXShikonin and its analogs inhibit cancer cell glycolysis by targeting tumor pyruvate kinase-M2Oncogene201130424297430610.1038/onc.2011.13721516121

[B108] GoldbergMSSharpPAPyruvate kinase M2-specific siRNA induces apoptosis and tumor regressionJ Exp Med2012209221722410.1084/jem.2011148722271574PMC3280873

[B109] Vander HeidenMGChristofkHRSchumanESubtelnyAOSharfiHHarlowEEXianJCantleyLCIdentification of small molecule inhibitors of pyruvate kinase M2Biochem Pharmacol20107981118112410.1016/j.bcp.2009.12.00320005212PMC2823991

[B110] LeACooperCRGouwAMDinavahiRMaitraADeckLMRoyerREVander JagtDLSemenzaGLDangCVInhibition of lactate dehydrogenase A induces oxidative stress and inhibits tumor progressionProc Natl Acad Sci U S A201010752037204210.1073/pnas.091443310720133848PMC2836706

[B111] ZhouMZhaoYDingYLiuHLiuZFodstadORikerAIKamarajugaddaSLuJOwenLBLedouxSPTanMWarburg effect in chemosensitivity: targeting lactate dehydrogenase-A re-sensitizes taxol-resistant cancer cells to taxolMol Cancer20109332014421510.1186/1476-4598-9-33PMC2829492

[B112] ColenCBShenYGhoddoussiFYuPFrancisTBKochBJMontereyMDGallowayMPSloanAEMathupalaSPMetabolic targeting of lactate efflux by malignant glioma inhibits invasiveness and induces necrosis: an in vivo studyNeoplasia20111376206322175065610.1593/neo.11134PMC3132848

[B113] LencioniRLoco-regional treatment of hepatocellular carcinomaHepatology201052276277310.1002/hep.2372520564355

[B114] GeschwindJFKoYHTorbensonMSMageeCPedersenPLNovel therapy for liver cancer: direct intraarterial injection of a potent inhibitor of ATP productionCancer Res200262143909391312124317

[B115] ValiMLiapiEKowalskiJHongKKhwajaATorbensonMSGeorgiadesCGeschwindJFIntraarterial therapy with a new potent inhibitor of tumor metabolism (3-bromopyruvate): identification of therapeutic dose and method of injection in an animal model of liver cancerJ Vasc Interv Radiol2007181 Pt 1951011729670910.1016/j.jvir.2006.10.019

[B116] ValiMVossenJABuijsMEnglesJMLiapiEVenturaVPKhwajaAAcha-NgwodoOShanmugasundaramGSyedLWahlRLGeschwindJFTargeting of VX2 rabbit liver tumor by selective delivery of 3-bromopyruvate: a biodistribution and survival studyJ Pharmacol Exp Ther20083271323710.1124/jpet.108.14109318591216PMC2760588

[B117] BirsoyKWangTPossematoRYilmazOHKochCEChenWWHutchinsAWGultekinYPetersonTRCaretteJEBrummelkampTRClishCBSabatiniDMMCT1-mediated transport of a toxic molecule is an effective strategy for targeting glycolytic tumorsNat Genet20134511041082320212910.1038/ng.2471PMC3530647

[B118] CaoXBloomstonMZhangTFrankelWLJiaGWangBHallNCKochRMChengHKnoppMVSunDSynergistic antipancreatic tumor effect by simultaneously targeting hypoxic cancer cells with HSP90 inhibitor and glycolysis inhibitorClin Cancer Res20081461831183910.1158/1078-0432.CCR-07-160718347186

[B119] FilomeniGCardaciSDa Costa FerreiraAMRotilioGCirioloMRMetabolic oxidative stress elicited by the copper(II) complex [Cu(isaepy)2] triggers apoptosis in SH-SY5Y cells through the induction of the AMP-activated protein kinase/p38MAPK/p53 signalling axis: evidence for a combined use with 3-bromopyruvate in neuroblastoma treatmentBiochem J2011437344345310.1042/BJ2011051021548882

[B120] NakanoATsujiDMikiHCuiQEl SayedSMIkegameAOdaAAmouHNakamuraSHaradaTFujiiSKagawaKTakeuchiKSakaiAOzakiSOkanoKNakamuraTItohKMatsumotoTAbeMGlycolysis inhibition inactivates ABC transporters to restore drug sensitivity in malignant cellsPLoS One2011611e2722210.1371/journal.pone.002722222073292PMC3206937

[B121] BeneteauMZuninoBJacquinMAMeynetOChicheJPradelliLAMarchettiSCornilleACarlesMRicciJECombination of glycolysis inhibition with chemotherapy results in an antitumor immune responseProc Natl Acad Sci U S A201210949200712007610.1073/pnas.120636010923169636PMC3523878

